This article has been retracted.

# Effect of Continuous Nutrition Management Intervention on Nutritional Status and Development of Premature Infants Based on Mobile Medical APP

**DOI:** 10.1155/2022/8586355

**Published:** 2022-08-08

**Authors:** Qing Zhang, Zhiyan Huo

**Affiliations:** Pediatrics Xingyuan Hospital, Yulin City, Shaanxi Province 719000, China

## Abstract

**Objective:**

To explore the effect of continuous nutrition management intervention based on mobile medical APP on the nutritional status and development of premature infants.

**Methods:**

Eighty premature infants treated in our hospital from May 2019 to April 2021 were enrolled. The patients were randomly divided into the control group and research group. The control group received routine nursing, and the research group received continuous nutrition management intervention based on mobile medical APP. The Neonatal Behavioral Neurological Assessment (NBNA) score, pain score, height, weight, head circumference, intellectual development score, serum Prealbumin (PA), retinol-binding protein (RBP), and disease occurrence were elucidated.

**Results:**

First of all, the NBNA scores of the two groups were compared. The behavioral ability, passive muscle tension, active muscle tension, original reflex, and general evaluation scores of the research group were significantly higher when compared to the control. Secondly, we compared the pain scores of the two groups, there was no significant difference between the two groups before nursing (*P* > 0.05), but the pain scores of the research group were lower compared to the control group during the period of blood collection, recovery, discharge, and 6 months after discharge (*P* < 0.05). Compared with the growth and development indexes of the two groups, there was no significant difference between the two groups before nursing (*P* > 0.05). After nursing, the GDS score of the two groups increased, and the GDS score of the research group was higher than that of the control group. The difference of data was statistically significant (*P* < 0.05). Compared with the motor scores of the two groups, there was no significant difference between the two groups before nursing (*P* > 0.05). After nursing, the motor scores of the two groups increased, and the scores of PDMS-2 and TIMP in the research group were higher than those in the control group, and the difference was statistically significant (*P* < 0.05). There was no significant difference in serum PA and RBP before nursing, but the serum PA and RBP in the two groups increased after nursing, and the PA and RBP in the research group were higher than those in the control group, and the difference was statistically significant (*P* < 0.05). Finally, we compared the incidence of diseases between the two groups. Before nursing, the incidence of infection, retinopathy, chronic lung injury and anemia in the research group was lower, when compared to the control, and the difference was statistically significant (*P* < 0.05).

**Conclusion:**

The intervention strategy of continuous nutrition management based on mobile medical APP for premature infants can significantly strengthen their nutritional status after discharge, promote their growth and development, improve their nutritional status, reduce the incidence of diseases in premature infants, and then enhance their quality of life.

## 1. Introduction

Premature infants refer to newborns whose gestational age is less than 37 weeks, some of their organs are immature, their nutritional status is low, and their adaptability is worse than that of full-term infants [1]. According to the global report on premature infants released by the World Health Organization (WHO), the global incidence of preterm births is more than 10%, and about 15 million premature babies are born every year [2]. China accounts for 7.8% of global preterm births, and about 1.2 million premature babies are born every year, making it the second largest country of preterm births after India. In recent years, with the development of assisted reproductive technology and the increase of elderly parturients and multiple pregnancies, the incidence of preterm delivery is showing a more severe upward trend [2]. Premature complications were the leading cause of death among children under the age of 5 worldwide in 2015, representing about 16 per cent of all deaths and 35 per cent of newborn deaths [3]. Fortunately, advances in perinatal medicine and neonatal intensive care technology have significantly improved the survival rate of premature infants, even at 22 weeks of gestational age. The survival rate is now 23.1% [4]. However, survivors had a high incidence of neurological disorders, with about 5% of premature infants diagnosed with cerebral palsy at a later stage, 35% with behavioral problems, and 26% with socioemotional incompetence [5]. For premature infants, if they are not given active nutritional support and special care, they are prone to complications such as growth retardation and infectious diseases, which will affect their intelligence, physique and neurological development, and even die in serious cases. Timely and effective intervention measures for premature infants can avoid the death of premature infants [5]. The nursing of premature infants acts as a long-term and continuous process, which is mainly borne by the family, but most guardians lack understanding of the nutritional needs and physiological development characteristics of premature infants, so they cannot provide scientific nutrition management for premature infants [6]. Although some of the problems can be solved by regular follow-up, there are still some problems, such as high prevalence rate of premature infants, many sequelae, and easy to lose follow-up [6].

In recent years, with the rapid development of mobile communication technology, Internet technology, and the increasing popularity of intelligent electronic devices, mobile medicine (MHealth) has been involved in all fields of medical rehabilitation and health care, and medical staff and patients are more and more receptive to Internet ideas and methods [7]. MHealth [7] refers to the practice of applying mobile devices such as mobile phones and patient monitoring devices in the fields of medicine and public health care. With the change of disease mode and medical service model, MHealth care has maintained a hot development trend and become the focus of research in our country [8]. The main forms of MHealth include smartphone information services and voice and mobile phone applications (APP), which are not limited by time and space, and have the advantages of convenient carrying, wide application, and timely feedback [8]. It provides a new way to realize doctor-patient interaction, health management, chronic disease surveillance, peer support, and so on. MHealth APP refers to the third-party applications of smartphones based on different operating systems to provide users with a variety of health-related information and services. The theoretical model and service content of continuous care based on MHealth APP for patients with chronic diseases are different. Yao and others have confirmed the applicability of “Internet + continuous nursing” guided by planned behavior theory in autistic children. Domestic scholars have applied the software based on technical acceptance model in stress injury management, and its effectiveness and feasibility of the promotion scheme have been proved [9]. Liu and others answered questions online by a multidisciplinary team composed of nursing experts and general practitioners [10], and Vogl et al. employed mobile applications to record the physiological status and health behavior of COPD patients [11]. Menke and others have pointed out that smartphones have a positive impact on extended care and can promote changes in the health care system [12]. With the popularity of smartphones, MHealth APP have been reported to be used to provide mobile medical services for patients with diabetes and essential hypertension with remarkable results [11]. At present, MHealth APP is mostly employed in maternal health management, but there is no research on continuous nutrition management intervention in premature infants. The purpose of this study is to analyze the effect of continuous nutrition management intervention with MHealth APP after discharge of premature infants, in order to provide reference for improving the effect of nutrition management of premature infants. The research results are reported as follows.

## 2. Patients and Methods

### 2.1. Patient General Information

Eighty premature infants treated in our hospital from May 2019, to April 2021 were enrolled. The patients were randomly divided into the control group and research group. The control group received routine nursing, and the research group received continuous nutrition management intervention based on mobile medical APP. In the control group, there were 23 males and 17 females, the gestational age was 31.85 ± 3.21 weeks (28-35 weeks), and the birth weight was 1454.23 ± 150.38 g (1260-1600 g). In the research group, there were 22 males and 18 females, the gestational age was 31.56 ± 3.33 weeks (28-36 weeks), and the birth weight was 1455.55 ± 150.64 g (1260-1600 g). There was no statistical significance in the general data of the two groups.

Inclusion criteria are as follows: premature infants: (1) gestational age 31-33 weeks, (2) birth weight ≥ 1500 g, (3) singletons or twins, (4) hemodynamic stability, and (5) at least 4 heel blood samples are expected to be collected within weeks; mother: (1) age ≥ 18 years old, (2) agree to participate in this study and sign informed consent form, and (3) have good communication skills.

Exclusion criteria are as follows: premature infants: (1) suffering from severe congenital diseases or deformities; (2) suffering from nervous system diseases or obvious nervous system symptoms; (3) using analgesics, sedatives, or muscle relaxants within 24 hours before outcome measurement; (4) need intubation and mechanical ventilation; and (5) heel tissue damage or inflammatory signals and mother: (1) reemployed to participate in this study and (2) critical condition, infectious disease, or mental illness.

Elimination and shedding criteria are as follows: (1) termination of kangaroo care due to mother or family reasons, (2) kangaroo care should not be continued due to serious changes in illness during the test, and (3) discharge, transfer, or death during the trial.

### 2.2. Nursing and Treatment Methods

The control group received routine treatment and nursing according to the guidelines for the management of premature infants [13], including warmth, respiratory management, nutritional support, prevention of infection, keeping blood glucose stable, maintaining electrolyte balance, and prevention and treatment of brain injury.

The research group received continuous nutrition management intervention based on mobile medical APP and adopted APP (Guangzhou Pushenmei Business Consulting Co., Ltd.) to carry out nutrition intervention. The specific measures are as follows. (1) One day before the discharge of the premature infant, the responsible nurse instructed the premature infant guardian to download for free through the smart phone, register the excellent doctor next to the APP, and instructed the premature infant guardian to log on to the APP to communicate with the doctor in real time, and to establish the premature infant mobile medical APP file database and so on. (2) Health education: the guardians of premature infants were drawn into the follow-up group of guardians of premature infants by responsible nurses. Every day, the responsible nurses sent in the follow-up group about the high-risk factors affecting the physical and neurological development of premature infants, and matters needing attention in the nursing process of premature infants, as well as the prevention and treatment of common concomitant diseases, milk powder feeding knowledge of premature infants, supplementary food knowledge and feeding emphasis, and other related contents. Guardians can also consult the popular science articles on nutrition management of premature infants published by clinicians through the APP moments and receive relevant guidance. Clinicians carry out health education related to nutritional management of premature infants through group follow-up notices, intragroup communication and guidance, online seminars, remote microclasses, and video explanations. (3) Feeding guidance: clinicians communicate with the guardians of premature infants through the APP chat interface to know the situation of premature infants in real time and then give timely guidance, and through the APP, it is suggested that the guardians of premature infants begin to supplement vitamin D to premature infants about 2 weeks after birth. (4) Data record: every month, the APP regularly prompts the guardian of premature infants to measure the growth and development indexes such as height, weight and head circumference of premature infants and records them in the data archives of the APP, so that the nurses in charge can monitor the growth and development of premature infants in real time. If the growth and development of premature infants is slow, the guardian can contact the medical staff for help at any time through the APP, and the medical staff can also use the APP to guide the guardian to adjust the nutritional support program in time and supervise its implementation. (5) Clinical early warning: after discharge, the guardian monitored the clinical early warning indexes of premature infants, such as cyanosis, body temperature not rising, fever, feeding intolerance, feeding difficulty, pallor of skin and nail bed, poor weight gain, diarrhea, night terrors, and sweating, like shaking the head, and occipital baldness. These indexes were set as the long-term notice in the follow-up group of the APP. If the above clinical early warning indicators appear in premature infants, it is suggested that guardians should use the APP for prehospital consultation, visual diagnosis, picture and text collection, video recording, medical history collection, and so on. If the clinical early warning of premature infants is only a simple problem, the nurse in charge will guide the guardian to solve the problem online through the APP. If it is a difficult, complex, or critical problem, then instruct the guardian to bring the premature infant to our hospital in time to make an appointment. Six guidance of intelligence and physical intervention: through the APP chat interface, the guardians of premature infants were followed up regularly every month, and the guardians were instructed to conduct early intellectual and physical intervention training for premature infants. Intelligence training includes visual, auditory, and tactile stimulation in the awake state of premature infants, as well as language and cognitive development training, such as listening to music, eye contact, giving fresh toys, and guiding speech. According to the age and physical development of premature infants, physical training should be carried out, such as baby exercises, hydrotherapy, looking up, turning over, climbing, and sitting. For the premature infants in the control group, routine telephone follow-up was employed for nutrition intervention. The health records of premature infants were established by responsible nurses. Fixed telephone follow-up once a month, conducted by the same instructor as the research group, to understand the growth and development, nutritional support, and disease occurrence of premature infants, and record the follow-up results of premature infants in their health records, and according to the individual situation of premature infants, guide the guardian to manage the body temperature, skin, nutrition and personal hygiene of premature infants. Two groups of premature infants were followed up for 6 months after discharge.

### 2.3. Observation Index

#### 2.3.1. Neonatal Behavioral Neurological Assessment

Neonatal Behavioral Neurological Assessment (NBNA) [14] was established by Professor Bao Xiulan on the basis of American Brazelton Neonatal Behavioral scoring method and French Amiel-Tison Neuromotor Test, combined with her own experience. This method can be employed to reflect the brain development of premature infants, and its prognostic value is better than that of cranial ultrasound and CT. The sensitivity and specificity of NBNA for brain development at postnatal day 7 were 88.9% and 82.6%, respectively, and the sensitivity and specificity for brain development at postnatal day 12-14 were 84.6% and 97.4%, respectively [15]. NBNA consists of 20 assessment items, which are assigned into 5 parts: behavioral ability (6 items), passive muscle tone (4 items), active muscle tension (4 items), primitive reflex (3 items), and general assessment (3 items). Each score has 3 grades, that is, 0, 1, and 2, and the total score is 40. The higher the score, the better the behavioral nerve development.

#### 2.3.2. Pain Score of Premature Infants

The pain score scale of preterm infants (PIPP) [16] is a comprehensive pain scale specially designed by the universities of Toronto and McGill in Canada according to the characteristics of premature infants. The specific contents of the assessment included seven items: heart rate, blood oxygen saturation, three kinds of facial activity (frowning, winking, and deepening of nasolabial sulcus), gestational age, and behavioral status (sleep or awakening). The score of each item is 0-3, the total score is the sum of 7 items, the lowest score is 0, the highest score is 21, the total score ≤ 6 indicates little/no pain, 7-12 indicates moderate pain, and >12 indicates severe pain. Cronbach's *α* coefficient of the scale was 0.72.

#### 2.3.3. Growth and Development Index

(Griffiths) the evaluation content of the Chinese version of the Development Assessment scale (GDS-C): GDS-C includes six areas: field A: sports: up and down the stairs, playing football, cycling, trotting and jumping, etc. Area B: personal-social: the ability to wear and undress, use cutlery, and use knowledge and information, such as whether you know your birthday or address, etc. Area C: language: say the color and name of the object, repeat words, describe a picture and answer a series of questions about the similarities/differences of the content, etc. Area D: hand-eye coordination: string beads, cut with scissors, copy graphics, write letters and numbers, etc. Area E: performance: building bridges or stairs, completing puzzles and modeling, etc. Field F: practical reasoning: items tested: count, compare size, shape, height. This field also tests children's understanding of dates, visual sorting ability, and understanding of right, wrong and right. A total of 100 points, less than 10 points indicate no progress, 10-20 points indicate average progress, and >20 points indicate obvious progress.

#### 2.3.4. Sports Evaluation

Exercise evaluation: PDMS-2 evaluation, that is, one evaluation before training and one month after training. The evaluation activity is carried out by a professional physician who is certified by the evaluation, and the guardian assists the baby to respond. Among them, the infants under 2 years old need to be corrected by age, and the infants under 2 years old should be evaluated in the later stage according to the corrected age. The specific evaluation items are as follows: in the evaluation of gross motor function of children, infants under 12 months of age need to test reflex (8 items), movement (89 items), and posture (30 items). The measured energy areas of children aged 1 to 6 years old were posture (30 items), movement (89 items), and physical manipulation (24 items). In the evaluation of fine motor function in children, grasping (26 items) and visual motor integration (72 items) were needed.

Evaluation of TIMP scale: all the evaluators who participated in the study were trained by the simplified Chinese version of the copyright and obtained the intermediate application qualification of the simplified Chinese version of the Infant Sports Performance Test. The evaluation process is carried out in the crib to ensure that the room is quiet, bright and warm, and the baby should be quiet and awake. TIMP consists of 42 items with a total score of 142. It is divided into two parts: observation items and induced items. The observation items included 1-13 items, and the performances of head control, limb movement, and restless movement were observed. If there is a corresponding performance, the score of each item is 1 point, and the score of nonappearance is 0. The evoked items included 14-42 items, and the infants were evaluated for head control, audio-visual stimulation response, limb and trunk movement, and defense action response in all postures, and the score range was 0-6 points. Some items (item 19/20, item 23/24, item 28/29, item 30/31, item 38/39, and item 41/42) are scored on the left and right sides, respectively.

#### 2.3.5. Nutrition Index

Nutritional index: 3 ml was collected from plantar venous blood of premature infants in the morning and placed in an anticoagulant tube of ethylenediamine tetraacetic acid. After 10 min was centrifuged with 2500 r/min (centrifugal radius as 5.5 cm) at 4°C, the supernatant was retained. The levels of serum prealbumin (PA) and retinol binding protein (RBP) were measured by BayerAdvia2400 automatic biochemical analyzer (Bayer Company, Germany).

#### 2.3.6. Incidence of Diseases in Premature Infants

Incidence of diseases in premature infants: the incidence of diseases in premature infants was recorded during the 6-month follow-up. The incidence of diseases in premature infants (%) = the number of cases of diseases in premature infants/the total number of cases of premature infants × 100%.

### 2.4. Statistical Analysis

SPSS 21.0 statistical software was employed to analyze the data of this study. Size software was employed to determine the minimum sample size to meet the statistical test of this study. The measurement data with normal distribution were expressed as $\bar{x}\pm s$, and the group *t*-test was employed to compare the two groups. For the counting data, the percentage (%) was employed to express, and the *χ*^2^ test was employed to compare the two groups. Bilateral test was employed in all statistical tests, and *P* < 0.05 indicated that the difference was statistically significant.

## 3. Results

### 3.1. NBNA Score Comparison

First of all, the NBNA scores of the two groups were compared. The behavioral ability, passive muscle tension, active muscle tension, original reflex, and general evaluation scores of the research group were significantly higher than those of the control group, and the difference was statistically significant (*P* < 0.05). All the data results are illustrated in Table 1.

### 3.2. Pain Score Comparison

Secondly, we compared the pain scores of the two groups, there existed no significant difference between the two groups before nursing (*P* > 0.05), but the pain scores of blood collection, recovery, discharge, and 6 months after discharge in the research group were lower than those in the control group, and the difference was statistically significant (*P* < 0.05). All the data results are illustrated in Table 2.

### 3.3. Comparison of Growth and Development Indexes

Secondly, we compared the growth and development indexes of the two groups. Before nursing, there was no significant difference between the two groups (*P* > 0.05). After nursing, the GDS score of the two groups increased, and the GDS score of the research group was higher than that of the control group, and the difference was statistically significant (*P* < 0.05). All the data results are shown in Table 3.

### 3.4. Sports Score Comparison

Secondly, we compared the motor scores of the two groups. Before nursing, there was no significant difference between the two groups (*P* > 0.05). The motor scores of the two groups were increased after nursing, and the PDMS-2 and TIMP scores of the research group after nursing were higher than those of the control group; the difference was statistically significant (*P* < 0.05). All the data results are shown in Table 4.

### 3.5. Comparison of Serum PA and RBP Indexes

Then, we compared the serum PA and RBP indexes of the two groups; there existed no significant difference before nursing, but after nursing, the serum PA and RBP indexes of the two groups increased, and the serum PA and RBP indexes of the research group were higher compared to the control, and the difference was statistically significant (*P* < 0.05). The results of all the data are illustrated in Table 5.

### 3.6. Comparison of Disease Occurrence

Finally, we compared the incidence of diseases. Before nursing, the incidence of infection, retinopathy, chronic lung injury, and anemia in the research group was lower compared to the control, and the difference was statistically significant (*P* < 0.05). All the data results are illustrated in Table 6.

## 4. Discussion

From 2000 to 2014, the global incidence of preterm birth increased from 9.8% to 10.6% [18]. With the progress of obstetrics and neonatal intensive care technology, the mortality of premature infants has decreased significantly, but the incidence is still very high [18]. Compared with full-term infants, premature infants show more school-related problems, poor cognitive ability and academic achievement in childhood, and lower educational level and socioeconomic achievements in adulthood [19]. With the change of social environment and economy, as well as the implementation of the three-child policy in China, the incidence of premature infants is increasing [19]. Due to the premature separation from the mother, brain hypoplasia, and hypoplasia of important organs, premature infants are prone to problems such as dystonia, growth retardation, and intellectual abnormality, which bring heavy burden to the family and society. It is reported that preterm delivery is an independent risk factor for abnormal physical and intellectual development in childhood, and the smaller the gestational age, the greater the adverse effect on the development of premature infants [18]. Therefore, the early nutrition management of premature infants is the key to improve the quality of life of premature infants. The American Academy of Pediatrics put forward the “high-risk infant-family-care” model, that is, the discharge of premature infants does not mean the end of nutritional intervention, but the beginning of a new nutritional intervention model [20]. Nutrition management intervention of premature infants is a long-term and continuous process, and regular follow-up after discharge is the focus to ensure the normal development of premature infants. However, the follow-up of premature infants after discharge is affected by guardian compliance, education level, economic level, population mobility, regional, and other factors, and the clinical follow-up rate is high [19]. With the widespread use of smart phones, MHealth has become a research hotspot in the field of medical and health. MHealth treatment refers to the use of portable, small communication devices, or third-party applications in wireless computers to meet the health information services of doctors and patients [20]. Although the premature infants are affected by congenital factors and their development is relatively poor, they have great growth potential, especially under 1 year old [17]. Therefore, early scientific nutrition intervention, reasonable supplement, and timely vitamin supplement for premature infants are helpful for them to obtain adequate nutrition, catch up with growth quickly, and shorten the development gap between full-term infants and full-term infants [21].

According to the results of this study, the scores of behavior ability, passive muscle tension, active muscle tension, primitive reflex, and general evaluation in the research group were significantly higher compared the control (*P* < 0.05). As such, the change of the research group was more significant and had better behavioral nerve performance, which was mainly reflected in behavioral ability, passive muscle tension and active muscle tension. Our conclusion confirms the promoting effect of continuous nutrition management intervention based on mobile medical APP on the behavioral nerve development of premature infants. In the study of Buhimschi et al. through the Neonatal Behavioral Assessment scale (NBAS), it was found that preterm infants from 31 to 33 weeks of age had better adaptation to visual and auditory stimuli and better directional response to external stimuli than newborns who received traditional nursing care after one hour of SSC with their mothers at the corrected gestational age of 37 weeks [22]. A study in Brazil employed the Neonatal intensive Care Unit Network Neurobehavioral scale (NNNS) to evaluate the effect of continuous nutrition management interventions based on mobile medical APP on correcting preterm infants of 36-41 weeks of gestational age and found that continuous nutrition management interventions based on mobile medical APP were associated with better state control, exercise quality, greater adaptability, and lower stress performance [23]. Although the behavioral neurological assessment tools employed in different studies are different, the conclusions support that the continuous nutrition management intervention based on mobile medical APP can promote the behavioral neurological development of premature infants. Preterm infants exposed to pain-related stress repeatedly have poor cognitive, motor, and behavioral nerve development, which is related to the changes of brain volume, brain structure, and function [24]. Although drug intervention may be a logical solution for pain relief, it is inappropriate and impractical to use it to relieve repeated operational pain in newborns, such as heel blood collection. It is reported that long-term repeated use of opioid analgesics can hinder the cognitive development of newborns at school age [25–27]. In this study, continuous nutrition management intervention based on mobile medical APP was used as an analgesic scheme in the process of repeated heel blood collection in premature infants. The results indicated that the analgesic effect of continuous nutrition management intervention based on mobile medical APP remained stable in the process of repeated pain. Compared with conventional nursing, continuous nutrition management intervention based on mobile medical APP can significantly reduce PIPP scores in blood collection and recovery period. This is also consistent with the findings of a recent foreign study, supporting the use of continuous nutrition management interventions based on mobile medical APP to relieve recurrent operational pain in premature infants [28, 29].

Prealbumin (PA) is a protein synthesized and secreted by parenchyma cells of liver, choroid plexus of brain, pineal gland, and so on. It has high sensitivity in reflecting malnutrition [30]. Retinol-binding protein (RBP), a transporter of vitamins in the blood, is synthesized by the liver and is an indicator of malnutrition [30]. Through the chat function of APP next to the excellent doctor, the responsible nurse and clinician can communicate with the premature infant guardian in real time and guide the guardian to make individual feeding plan according to the development of premature infant, so as to ensure the high quality and comprehensive nutrition of premature infant [31]. The results of this study indicated that after intervention, the serum levels of PA and RBP in the research group were significantly higher compared to the control (*P* < 0.05). The results indicated that the nutritional level of premature infants in the research group was significantly improved, and after intervention, the height, head circumference, and weight of premature infants in the research group were significantly better than when compared to the control group (*P* < 0.05). It can be noticed that the premature infants in the research group have good physical development, and the nutrition management intervention based on mobile medical APP strategy can effectively improve their nutritional level and promote their physical development. The results of this study also showed that after the intervention, the scores of intelligence scale and exercise scale of premature infants in the research group were significantly higher than those in the control group (*P* < 0.05). This shows that the intellectual development and motor ability of premature infants in the research group are better. Based on mobile medical APP, the intervention training of premature infants' intelligence and physique can effectively promote the intellectual development of premature infants, in order to set clinical early warning indicators next to APP, such as blue complexion, low body temperature, fever, feeding intolerance, feeding difficulties, pallor of skin and nail bed, poor weight gain, diarrhea, night terrors, and sweating, like shaking head and occipital alopecia. In this study, the results of 6-month follow-up of the two groups of premature infants indicated that the incidence of premature infants in the research group was significantly lower compared with the control group (*P* < 0.05). It is suggested that the utilization of mobile medical APP for nutritional intervention of premature infants and the setting of clinical early warning indicators can effectively reduce the incidence of diseases in premature infants. Nutrition management intervention of premature infants based on mobile medical APP can significantly improve the nutritional status of premature infants after discharge, promote their growth and development, reduce the occurrence of premature diseases, and then improve the quality of life of premature infants [31]. Our study still has some shortcomings. Firstly, the quality of this study is limited due to the small sample size we included in the study. Secondly, this research is a single-center study and our findings are subject to some degree of bias. Therefore, our results may differ from those of large-scale multicenter studies from other academic institutes. Our research is still clinically significant and further in-depth investigations will be carried out in the future.

In conclusion, the continuous nutrition management intervention strategy of preterm infants based on mobile medical APP can significantly improve the nutritional status of premature infants after discharge, promote their growth and development, enhance their nutritional status, reduce the incidence of diseases in premature infants, and then improve their quality of life.

## Figures and Tables

**Table 1:** Comparison of NBNA scores between the two groups ($\bar{x}\pm s$, points).

Grouping	*N*	Capacity	Passive muscle tension	Active muscle tension	Original reflection	General assessment
Control group	40	8.18 ± 0.53	6.42 ± 0.75	5.21 ± 0.53	5.07 ± 0.66	5.44 ± 0.15
Research group	40	9.48 ± 0.42	7.59 ± 0.31	5.82 ± 0.33	5.67 ± 0.31	5.92 ± 0.12
*t*		12.158	9.118	6.179	5.204	15.803
*P*		0.000	0.000	0.000	0.000	0.000

**Table 2:** Comparison of pain scores between the two groups ($\bar{x}\pm s$, points).

Grouping	*N*	Before nursing	Blood collection period	Recovery period	When discharged from the hospital	6 months after discharge
Control group	40	3.51 ± 0.21	14.59 ± 1.21	10.85 ± 1.22	5.84 ± 0.41	3.11 ± 0.26
Research group	40	3.48 ± 0.23	13.28 ± 1.34	9.86 ± 1.62	4.78 ± 0.44	1.93 ± 0.11
*t*		0.609	4.588	3.087	11.147	26.435
*P*		0.544	0.000	0.000	0.000	0.000

**Table 3:** Comparison of growth and development indexes between the two groups ($\bar{x}\pm s$).

Grouping	*N*	GDS	
		Before nursing	After nursing
Control group	40	57.93 ± 4.21	82.39 ± 3.44
Research group	40	57.69 ± 4.41	90.92 ± 1.55
*t*		0.248	14.298
*P*		0.804	0.000

**Table 4:** Comparison of intellectual development scores between the two groups ($\bar{x}\pm s$, points).

Grouping	*N*	PDMS-2		TIMP	
		Before nursing	After nursing	Before nursing	After nursing
Control group	40	80.83 ± 3.55	83.77 ± 3.31	49.95 ± 3.12	68.92 ± 3.31
Research group	40	80.39 ± 3.45	90.95 ± 3.31	49.69 ± 3.45	80.81 ± 2.53
*t*		0.562	9.700	0.353	18.049
*P*		0.575	0.000	0.724	0.000

**Table 5:** Comparison of serum PA and RBP indexes between the two groups ($\bar{x}\pm s$).

Grouping	*N*	PA(mg/L)		RBP(mg/L)	
		Before nursing	After nursing	Before nursing	After nursing
Control group	40	90.95 ± 4.11	120.91 ± 4.66	103.96 ± 10.21	128.82 ± 13.31
Research group	40	90.58 ± 4.12	138.94 ± 7.45	103.83 ± 10.53	140.82 ± 12.85
*t*		0.402	12.976	0.056	4.102
*P*		0.688	0.000	0.955	0.000

**Table 6:** Comparison of disease occurrence between two groups of children (*n* (%)).

Grouping	*N*	Infected	Retinopathy	Chronic lung injury	Anemia	Total incidence rate
Control group	40	4 (10.00)	5 (12.50)	2 (5.00)	5 (12.50)	16 (40.00)
Research group	40	1 (2.50)	1 (2.50)	1 (2.50)	1 (2.50)	4 (10.00)
*χ* ^2^						9.600
*P*						0.001

## Data Availability

The datasets used and analyzed during the current study are available from the corresponding author upon reasonable request.
